The article "Environment-Friendly Vocal Music Ecological Education: Sustainable Development of Vocal Music Education from the Perspective of Building" was published in 2022. Journal: J Environ Public Health.

# Environment-Friendly Vocal Music Ecological Education: Sustainable Development of Vocal Music Education from the Perspective of Building

**DOI:** 10.1155/2022/5168389

**Published:** 2022-08-23

**Authors:** Gengyuan Zhang

**Affiliations:** Xinxiang University, Xinxiang 453003, China

## Abstract

With the acceleration of the modernization of human society, natural ecology is continuously destroyed, which inevitably brings about the crisis of the human spirit, and human beings progressively lose the ability to draw power from nature. Similarly, music is losing its function of freeing people from secularity and becoming a carrier of pure utility. For a long time, there have been some disharmonious factors in the ecological environment of vocal music teaching. For example, some vocal music teaching facilities are out of date, vocal music course resources are single and scarce, vocal music courses are comparatively isolated and lack organic integration with other courses, and relevant art practices and scientific research activities of teachers and students are not carried out well after class, comprehensive quality of teachers cannot be effectively improved, and external communication of colleges and universities is not enough. This has affected the quality of vocal music teaching to a certain extent. Accordingly, an environment-friendly ecological vocal education emerged. In addition, both building and music are the supplement and creation of the human living environment by the material organization. Consequently, their performance has similar characteristics of origin. Thus, from the perspective of the building, we touch the music, listen to the building, and analyze the integration of ecological vocal music education and building. The empirical test verified the effect of ecological vocal music teaching under the building vision.

## 1. Introduction

As human civilization rapidly modernizes, natural ecology is continually destroyed. This leads to a crisis of the human spirit, and people lose their capacity to draw strength from nature over time [1, 2]. Similarly, the art of music is losing its function of freeing people from material and secular fetters and becoming a carrier of pure utility. The development of music art is inseparable from the objective existence of music function and people's deepening aesthetic understanding of it [3–5]. Therefore, music must reconstruct the overall function of music aesthetic education based on the original concept, guided by ecological philosophy and using the concept of ecological aesthetics for reference. Music ecology studies music aesthetic phenomenon and cultural practice from the perspective of ecology and ecological philosophy [6, 7]. This kind of research should pay attention to three levels of theoretical issues. First is music ecocriticism, whose task is to analyze the natural ecological thought and ecological holism contained in music works. Aesthetic ecocriticism aimed at music works has ecological characteristics, with a new definition of “vision fusion,” followed by the auditory ecological problem of music aesthetics. Music ecology should study the ecological environment in which music exists, the experiential changes caused by environmental changes, and the relationship between human auditory experience, sound form, and stage environment. With the development of ecology, the ecological rationality of music is also called to play the educational role of the integral function of music and grasp the living experience of human beings with ecological thinking and the meaning of life's existence in ecological survival.

Singing comprises three elements: singing skills, emotional expression, and scientific, humanistic spirit [8]. Taking the “bucket effect” as an analogy, each aspect of the singing art is a piece of wood board that makes up the bucket, which may be uneven. If we want to increase the capacity of the bucket, the only way is to repair the weakness and strengthen the strength. Similarly, a good singer must also weigh the relationship between various elements of singing, improve its strengths, and complement its weaknesses. Singing takes the human voice as the musical instrument, and the whole process of vocalization and singing is the whole process of creative imagination and artistic expression by adjusting the relevant vocal organs under the control of the higher nerves of the brain. Vocal music education is a fundamental part of music education [9, 10]. Driven by the current educational reform trend, vocal music education in the 21st century must be open, integrated, and high-quality art education, that is, ecological vocal music education. Ecological vocal music education differs from cramming vocal music education and gardening vocal music education.

Cramming vocal music education, namely, teacher-led vocal music education, is a kind of education to accelerate the training of professional talents to adapt to the industrialization trend [11]. The biggest drawback of this kind of education is that, as in industrial agriculture, it treats students as a kind of land to be developed, rather than as in ecological agriculture, which mainly develops the soil's natural fertility [12]. The heavy use of chemical fertilizers in industrial agriculture results in increased productivity, but the natural structure and fertility of the soil are destroyed, and the environment is polluted. Cramming vocal music education tries its best to cram students with knowledge of vocal music singing skills in the hope of rapidly developing students with rich singing skills [13, 14]. Nevertheless, the result is disastrous. Students may learn a lot of singing skills and knowledge. However, their psychological ecological structure is severely damaged, not only losing the ability to create but also polluting the whole learning environment. Taking specific vocal music teaching as an example, the teacher lets the students practice voicing, blindly forces the students to submit to imagination according to the way of thinking of the teacher, and takes some so-called correct sound position or expression form of the emotional mood of the song as the “model” which the students imitate, firmly holds the development space of students' vocal music singing, and receives and imitates it as the only way of vocal music teaching. Imagine that in this kind of atmosphere of vocal music class, the students' active singing, singing image perception, and artistic expression will be ruthlessly stifled.

Ecological vocal music education also surpasses gardening vocal music education. The gardening vocal music education is the opposite of cramming vocal music education, an educational form of students' independent development [15]. It draws on the concept of ecological restoration and holds that people must learn to respect and obey nature. There is a potential development of human beings, and the task of educators is to create conditions for the development of human potential, like a gardener, so that it can be developed in a predetermined process and grow naturally like a plant [16]. The fatal aspect of gardening education is that they see human potential as something already existing, like oil at the bottom of the sea that can burst out of itself once it breaks through the surface. The gardening vocal music education lays too much emphasis on students' independent and free development, which often empty the role of teachers, and their ability and potential cannot be brought into play. This view of education blindly allows students to figure it out by themselves; contrary to the basic aesthetic principles, students' singing and artistic treatment is excessively free and loose, and the “personality” is absolutized and naturalized and lacks proper guidance from teachers [17]. Frequently, it is a phenomenon that students deviate from a music score.

Different from cramming vocal music education and gardening vocal music education, ecological vocal music education holds that healthy art education is a kind of vocal music skill education and a more comprehensive and sustainable development of quality education [18, 19]. To sum up, ecological vocal music education is a dynamic and scientific system of “student-led and teacher-led.” Its core principles are as follows. (i) First is the linking humanistic and scientific consciousness of vocal music education. That is, vocal music education is integrated with the scientific teaching method and the spirit of scientific research. (ii) The teacher must decline from the teaching status. At the same time, the student must rise from the inactive status, and the two form an ecological relationship of mutual stimulation, improvement, complementarity, and mutual growth. Students are trained to master vocal skills and then actively express their feelings, forming their singing style. The main contribution of this paper is that the sustainable development of environment-friendly vocal music ecological education from the perspective of the building is studied.

The rest of the paper is structured as follows. In Section 2, the construction of environment-friendly ecological vocal music teaching is studied. Sustainable development of vocal music education from the perspective of the building is presented in Section 3.  Section 4 gives the discussion of this paper.

## 2. Construction of Environment-Friendly Ecological Vocal Music Teaching

The quality of vocal music teaching is closely related to the harmony of teaching ecological environment. High-quality vocal music teaching is inseparable from harmonious teaching ecological environment [20]. Colleges and universities should strengthen environment-friendly classroom construction, course construction, and environment-friendly scientific research construction. Furthermore, colleges and universities should comprehensively follow up on relevant supporting measures, optimize the quality of hardware resources, software resources, and human resources, and provide robust and reliable guarantee for the construction of an environment-friendly ecological vocal music teaching environment from a multichannel and all-round perspective, which are presented in the following aspects [21, 22].

### 2.1. Strengthening the Construction of Modern Vocal Music Teaching Facilities

Modern teaching facilities are the fundamental guarantee to realize environment-friendly ecological vocal music teaching. Otherwise, the modernization of teaching means is not feasible, and environment-friendly ecological vocal music teaching is out of the question. Colleges and universities should proceed from the teaching reality, according to the specific situation of students' classroom teaching and extracurricular practice, strengthening the construction of teaching facilities, such as upright piano, grand piano, multimedia classroom, MIDI classroom, concert hall, audio and video reference room, and professional recording studio [23, 24]. For example, the teacher can optimize classroom teaching through a computer-aided method and its powerful multitrack recording function. Various audio-visual materials can be made for students to learn after class and consolidate the teaching quality.

### 2.2. Accelerating the Exploitation of Multichannel Vocal Music Course Resources

To have a basis for the technical, artistic, and academic problems encountered in vocal music teaching, colleges and universities should actively develop and rationally use all kinds of curriculum resources in school [25]. For example, the vocal music teaching and research office should purchase music books, magazines, audio, and audio-visual materials. At the same time, colleges and universities should actively build the school library, such as electronic information retrieval system construction, to facilitate teachers and students to find all kinds of information. In addition, teachers should make extensive use of social resources such as libraries and museums outside the school as a beneficial supplement to the curriculum resources inside and outside the school to form environment-friendly curriculum resources inside and outside the school and improve the quality of vocal music teaching [26].

### 2.3. Promoting the Reform of Rationalization of Vocal Music-Related Courses

Vocal music course is not isolated, and other courses constitute a curriculum ecosystem related to each other, which should be environment-friendly [27]. Colleges and universities should carry out necessary vocal music curriculum reform, for example, setting up interdisciplinary educational courses (vocal music pedagogy, vocal music physiology, and vocal music psychology), broadening the primary curriculum (natural sciences, humanities, and social sciences), increasing electives (Chinese vocal art history, foreign vocal art history, Chinese and foreign art songs, and opera appreciation), integrating professional courses and strengthening the connection between professional disciplines (comprehensive vocal music course), and adding demonstration course. Through a series of rationalized vocal music-related course reforms, the teaching quality will be improved, and the students' cultural connotation, artistic accomplishment, and singing ability will be enhanced.

### 2.4. Carrying Out Multichannel Vocal Music Course Art Practice

The essence of vocal music art is a kind of practice, and vocal music teaching is also a kind of teaching of artistic practice. Therefore, to enable students to solve practical problems and improve efficiency, they should be taken part in practice in a variety of ways. The practice of vocal music should be actively expanded to extracurricular [28, 29]. For example, they hold class solo concerts, individual solo concerts, vocal performances, competitions, and lectures. Vocal music teachers should give positive guidance to students' artistic practice and encourage students to participate in artistic practice actively. Colleges and universities should include this work into teachers' workload, provide the necessary support, and guarantee related equipment, funds, and sites.

### 2.5. Establishing Interactive Vocal Music Course for Scientific Research Organization

Vocal music teaching is a technical, artistic, and academic organic unity. The three levels of vocal music theory include not only technical theory and artistic theory but also academic theory. Teachers should emphasize strengthening academic research, establish vocal music art research institutions, encourage students to participate in scientific research activities, create an overall academic atmosphere, and carry out academic activities widely [30]. The content, scope, and angle of the research group should be as rich and colorful as possible, such as the technique of vocal music, the analysis of vocal music works, the cultivation of vocal music performance, and the development and contrast of the styles of Chinese and foreign vocal music. In addition, local vocal music research can also be carried out to broaden the horizon of exploration. Through a series of scientific research activities, some problems have been studied more deeply and thoroughly after class. This not only improves teaching efficiency but also enables students to cultivate the spirit of scientific research, strengthen the ability of scientific research, improve the level of scientific research, and develop the potential of scientific research.

### 2.6. Carrying Out All-Round Vocal Music Teacher Quality Training

High-quality vocal music teachers are the core of constructing environment-friendly ecological vocal music teaching. At the same time, as the vocal music teachers' ongoing study, colleges and universities should also actively give guarantees and support and carry out all-around quality training for the teachers [31]. We should regularly invite famous vocal music performing artists and vocal music educators to guide colleges and universities, including academic lectures, symposia, concerts, and other forms, to ensure that teachers constantly renew their educational ideas, change their teaching ideas, and improve their professional level. In addition, colleges and universities should organize teachers to study in the vocal music department of the top music colleges and universities in China. In this way, teachers' humanistic, artistic, and professional quality will be comprehensively improved, thus providing continuous power and vitality for the further construction of environment-friendly ecological vocal music teaching. The construction of environment-friendly vocal music ecological education is shown in Figure 1.

The realization of the goal of constructing environment-friendly ecological vocal music teaching cannot be achieved without the coordination of teachers and students, as well as the strong support from colleges and universities in terms of venues, equipment, funds, and policies. We should start from the above aspects to maximize the construction of environmentally friendly factors so that the environment-friendly ecological vocal music teaching will show a thriving, vigorous, and beautiful situation and coruscate with infinite youthful vitality.

## 3. Sustainable Development of Vocal Music Education from the Perspective of the Building

Among the associations and comparisons between different art categories, the connection between building and music is perhaps the most often observed. When people approach buildings and listen to music, there is always some contrast, imagination, and feelings and thoughts. Friedrich Von Schelling also said, “Architecture in general is frozen music.” Both building and music are the supplement and creations of the human living environment by the material organization [32]. Therefore, their performance has similar characteristics of origin. The relationship between building and music is manifested in the aspects of language, structure, symbol, and dynamics. Whether in ancient times, in the baroque era, or today, the interaction between buildings and music always takes place around people.

### 3.1. Touching the Music

People experience music not only with their ears but also with their bodies. When sound reaches the ear in the whole frequency band, or when part of the vibration is transmitted through the building space, part of the frequency also shakes the body cavity. This is why deaf people can also dance to the rhythm of the music. Therefore, we can say that music's impact on people is all-around. We can also experience the part of the music only felt by the ear through headphones. If we compare this feeling with the music from the air and the room, there will be a significant disadvantage. In the case of an instrumentalist, the instrument's vibrations are transmitted directly to the body, bringing the player and the music closer together [33]. Building and musical instrument manufacturing are ergonomic in particular. Instruments are constantly developing and improving, and playing techniques are constantly enriching.

Touch the music means that music gives us impressions of sights, materials, and colors that can be felt visually, by touch, and by vibration. Touch the music, as an intuitive sense of sound image, comes more from the instruments and materials associated with the sound and the media associated with the harmonic environment. As the structure and rhythm of the music unfold, this intuition forms a sequence that shapes a beautiful auditory world. There is a type of bamboo ware ensemble performance in Chinese folk music [34]. In this performance, people can recognize the sounding instrument from all kinds of round, sharp, or coarse, broken sounds. This is because in life when using bamboo instruments and approaching the bamboo hut, we have already had the experience of hearing and hearing them together. In building, people do almost the same in visual and tactile spaces [35]. The rough and smooth materials in architectural expression may be associated with the alternation of male and female voices in vocal, the contrast between the high-pitched Qin opera and the poignant Yue Opera, or the combination of drum and flute sounds. The black and white configuration of the building may be associated with the violent beating of the rhythm or the appearance of rest in the music.

Building and music come from and are products of the universe's and nature's movement. However, in the different modes of motion, the experience of touch, motion, or vibration is a seemingly immobile but deeply moving phenomenon. The expression of building and music in this direction undoubtedly comes from their unique material origin, related to the symbols, dynamic sense, and psychological field of architectural music. In a word, the beauty of building and music permeates the vocal and physical experience.

### 3.2. Listening to the Building

Music is a moving thing. The singing of music is the process in which people produce music through specific material movement while the transmission of music, or the process of “listening to music,” is a transmission of the dynamic process. From physics, music is transformed from the operational movement of playing to the ringing vibration of instruments, that is, the ringing vibration of the instrument's pipe, string, or vibrating cavity, which transmits music to the audience through sound waves in space, triggering the listener's heart and feeling the dynamics of vocal music [36]. This is about the intuition of the beauty of musical movement. Similarly, building construction requires a lot of energy and power to process, shape, transport, lift, position, and assemble building materials and other weaving operations. The result of this operation process is solidified in the internal and external image of the building, and the resulting expression of the structure and form of the building is also full of rich, dynamic information. According to weaving, when we listen to music, we follow the weaving of vocal music with our hearts and ears. When we watch buildings, we follow the traces of architectural weaving with our eyes and body.

The beauty of music is the movement of music. When we relate the concept of the music field, the movement of music is not only the performance of music but also the movement of human consciousness following the music field. When listening to music, people hear only one or a few notes at each moment. Through memory, we accumulate all the notes of the moment and form a general impression of the music. In music, we cannot hold memories in any one moment, and our overall impression of the music synthesizes this dynamic memory. This following process is a synchronous process of predicting and expecting in time and space. It is suspense, anticipation, and anticipation of beauty or a dialogue between a favorite and familiar work. When observing and touring the building, the shape and space of the building unfold before the eyes. Fovea centralis is the only small area of sharp resolution in the human eye, which is a tiny patch about two degrees in the middle of the visual field. So when reading a book, scan the line by line, word by word. Moreover, because the eye moves so fast, we can build up a detailed image of the object we want to observe from the tiny flashes of vision. This is the process of people seeing a building, which is very similar to listening to music.

It can be seen that the beauty of music is the movement of human consciousness following the music field, and the beauty of the building is the movement of human consciousness and behavior following the construction field. With the imagination of movement and the experience of movement, we can feel the beauty of the building. Therefore, when we think about the relationship between building and music, we should try our best to regard the building as “dynamic art” rather than just “frozen music.”

### 3.3. Analysis of the Integration of Vocal Music Education and Building

Environment-friendly ecological vocal music education occupies an essential position in the current music teaching reform because of the current focus on promoting quality-oriented education. In order to improve students' comprehensive quality level, we must strengthen the development of comprehensive quality. Therefore, environment-friendly ecological vocal music education, as one of the contents of music education, has played an important role and has been paid more and more attention at the present stage. However, due to the influence of the exam-oriented education concept in the past, ecological vocal music teaching has not received due attention, so teaching methods and teaching content have not been improved to a certain extent [37]. From the perspective of the building, we discuss the integration between environment-friendly ecological vocal music education and building and the integration approach based on the correlation characteristics to promote the level of environment-friendly ecological vocal music education.

The relation between building and environment-friendly ecological vocal music education for the building is to reflect the idea of transforming nature and fully reflect the idea of harmonious coexistence and sustainable development between man and nature in the architectural design process. With the improvement of living standards and highly developed economy, the building is not only a place for daily living and entertainment but also gradually becomes an extension and entity embodiment of people's thoughts. Therefore, the high-level cultural connotation of the building must be reflected in the current building design ideas to improve the ideological nature of building design and increase the creativity of the content in the design process.

The building is a kind of art, compared with other types of art, with architectural style and technique characteristics that are essentially the construction of a mode of thinking. In building design, different views and ideas are included to fully interpret each building design idea and absorb the breakthrough and innovative ideas. Because of this, the building design is open and will give recognition and tolerance to any future ideas and concepts. It will also demonstrate and absorb for reference, which has reference value for any art form since the development of any art form needs continuous compatibility and innovation to achieve sustainable development.

In terms of environment-friendly ecological vocal music education, with the improvement of the requirements and level of music teaching, the content and methods of vocal music teaching should keep pace with the times so that students can be really attracted by the course content and learn knowledge at the same time and gradually improve themselves and enhance their character quality. Therefore, the traditional educational methods and ideas are not suitable at present. We need to learn from similar ideas and experiences to gradually improve the framework and methods of environment-friendly ecological vocal music education. In terms of environment-friendly ecological vocal music education and building, there are a lot of similarities between them in the form of art construction and expression [38, 39]. Suppose we focus on the characteristics of relevance. In that case, we can analyze the correlation and similarity between ecological vocal music education and building and find that they have common ground in three aspects: perceptual appreciation, emotional appreciation, and rational appreciation. In environment-friendly ecological vocal music education, corresponding teaching methods and modes can also be summarized based on these similarities. Through the ideological connotation of building design, the level of environmental-friendly ecological vocal music education can be improved so that students can learn vocal music more profoundly and experience the beauty of vocal music through comparison and correlation. Through in-depth analysis, we can find that there are similar characteristics between environment-friendly ecological vocal music and architecture in terms of construction form and rhythm and also in terms of appreciation of correlation. Therefore, it is practically feasible and basic to integrate architectural ideas into environment-friendly ecological vocal music education.

To sum up, for the current vocal music education, it is necessary to reform environment-friendly ecological vocal music education and reestablish educational goals in the new era to adapt to the reform requirements education from many aspects. It is feasible to improve the teaching level of environment-friendly ecological vocal music by integrating building thought into the education of environment-friendly ecological vocal music.

### 3.4. Empirical Test

In this paper, 100 students from the Music Department of Xinxiang University were selected as research objects. They were divided into a control group (group 1–group 5) and an experimental group (group 6–group 10). For fairness, put 100 students according to their grade point average ranking of the previous semester into groups 1 and 6, followed by groups 2 and 7, and so on, and the order within the group is random. The experimental group used an environment-friendly ecological vocal music teaching method, while the control group used the conventional teaching method. After a semester, we judge the effectiveness of environment-friendly ecological vocal music teaching from the building perspective by the vocalization indicators of students' hum resonance, breath, continuity of subinterval, staccato, practice above fifth, multivowel, extended range of multivowel, continuity of significant intervals, and extended range pulsation. In addition, we selected ten teachers majoring in vocal music in the music department to score students' vocalization and recorded the average scores. As seen in Table 1, the average score of the experimental group was higher than that of the control group, which was 13.31% higher on average. This also shows the effectiveness of environment-friendly ecological vocal music teaching from the perspective of the building. The teacher combines the environment-friendly ecological vocal music education with building, promotes each other in learning, interprets the connotation of building, and enables students to truly realize the correct building idea and the relationship between vocal music education and vocal music elements. Vocal music and building are interlinked in time and space, transforming into each other. In the process of integration, it is necessary to recognize the similarities between the transformation of the two to play with ease and improve the ability of environment-friendly ecological vocal music education.

## 4. Conclusion and Discussion

This paper studies the sustainable development of environment-friendly ecological vocal music education from the perspective of the building. In the process of exploring environment-friendly ecological vocal music education and the integration of building ideas, it is necessary to understand that although there are many similarities between vocal music and building, after all, they belong to different sensory art forms, so it is necessary to master the transformation between the two in the integration.

### 4.1. Familiarizing the Essence of Vocal Music

In environment-friendly ecological vocal music education, teachers must understand the essence of vocal music education and the essence of vocal music development and interpret it correctly for students. Because for most students, the initial understanding of vocal music is singing, although different notes can play different music, for the essence of vocal music and the role and value of vocal music, especially environmental-friendly ecological vocal music education, students do not particularly understand. To achieve better integration between environment-friendly ecological vocal music education and building ideas, students should understand the essential role of vocal music education and its impact on students' personal growth. Therefore, vocal music should be interpreted and explained from many aspects, such as singing skills and vocal exercises.

### 4.2. Understanding of Building Ideas

Building ideas are far from each other for students studying vocal music, but there are many things in common between building and vocal music if we look at the art form and the presentation and expression of art. Therefore, in order to make students better able to combine vocal music and building ideas to study and promote each other, it is necessary to interpret the connotation of building ideas so that students can truly realize what is the right building ideas, as well as the relationship between environment-friendly ecological vocal music education and music elements.

### 4.3. Key to Integration of Environment-Friendly Ecological Vocal Education and Building Ideas

The combination of different melodies and tunes in vocal music is just like the different structures and materials that constitute the building itself. The balanced collocation of building materials and structures constitutes a strong artistic architectural form while combining musical elements constitutes a fluid building. Therefore, vocal music and building have interoperability in time and space. In the integration process, we also need to recognize the commonality of conversion between them. In this way, we can be more skilled and not naturally practice the integration between the two, which does not affect students' vocal music learning.

To sum up, studying the sustainable development of environment-friendly ecological vocal music education from the building perspective is feasible and plays a far-reaching role in the current vocal music education work. It is necessary to do an excellent job in the integration and in-depth research between the two.

## Figures and Tables

**Figure 1:** Environment-friendly vocal music ecological education.

**Table 1:** Scoring of student vocal exercises.

		Hum resonance	Breath	Continuity of subinterval	Staccato	Practice above fifth	Multivowel	Extended range of multivowel	Continuity of major intervals	Extended range pulsation
Control group	Group 1	3.98	4.12	4.05	3.87	3.92	4.06	3.88	4.06	4.12
	Group 2	4.04	4.21	4.11	3.52	3.97	4.12	3.87	4.01	3.97
	Group 3	3.88	4.05	4.23	3.49	4.05	3.88	3.69	3.96	4.05
	Group 4	3.87	3.98	3.99	4.01	4.11	3.96	3.91	3.84	4.06
	Group 5	4.01	4.06	3.87	4.08	3.86	4.07	3.97	3.91	3.99

Experimental group	Group 6	4.75	4.78	4.65	4.81	4.67	4.75	4.39	4.45	4.62
	Group 7	4.78	4.51	4.51	4.83	4.51	4.39	4.21	4.38	4.37
	Group 8	4.65	4.63	4.52	4.64	4.66	4.54	4.29	4.51	4.57
	Group 9	4.81	4.74	4.67	4.51	4.48	4.68	4.51	4.25	4.59
	Group 10	4.74	4.66	4.73	4.67	4.76	4.55	4.44	4.63	4.46

## Data Availability

All data used to support the findings of the study are included within the article.
